This article has been retracted.

# Recent Advances in DENV Receptors

**DOI:** 10.1155/2013/684690

**Published:** 2013-04-23

**Authors:** Shuyu Fang, Yanhua Wu, Na Wu, Jing Zhang, Jing An

**Affiliations:** Department of Microbiology, School of Basic Medical Sciences, Capital Medical University, Beijing 100069, China

## Abstract

Dengue is an old disease caused by the mosquito-borne dengue viruses (DENVs), which have four antigenically distinct serotypes (DENV1–4). Infection by any of them can cause dengue fever (DF) and/or a more serious disease, that is, dengue hemorrhagic fever (DHF) or dengue shock syndrome (DSS). In recent decades, incidence of dengue disease has increased 30-fold, putting a third to half of the world's population living in dengue-endemic areas at high infection risk. However, the pathogenesis of the disease is still poorly understood. The virus binding with its host cell is not only a first and critical step in their replication cycle but also a key factor for the pathogenicity. In recent years, there have been significant advances in understanding interactions of DENVs with their target cells such as dendritic cells (DC), macrophages, endothelial cells, and hepatocytes. Although DENVs reportedly attach to a variety of receptors on these cells, consensus DENV receptors have not been defined. In this review, we summarize receptors for DENVs on different cells identified in recent years.

## 1. Introduction

Dengue viruses (DENVs) belong to the Flaviviridae family. Four antigenically distinct serotypes of the viruses (DENV1–4) are transmitted to humans through the mosquito vector, *Aedes aegypti*. In the last century, dengue has escalated in geographic distribution and disease severity and therefore becomes an important public health concern worldwide. According to reports of the World Health Organization (WHO), dengue disease is endemic in more than 100 countries in Africa, the Americas, the Eastern Mediterranean, Southeast Asia, and the Western Pacific. With South-East Asia and the Western Pacific the most seriously affected, approximately 500,000 people with DHF require hospitalization each year, of whom 2.5% die. 

DENVs are small (50 nm) enveloped particles with a single-stranded messenger (positive) sense RNA of approximately 11 kb in length. The single open reading frame is directly translated into a polyprotein precursor [1], which is subsequently glycosylated by cellular glycosyltransferases and cleaved by proteases from virus and host cell to release three structural proteins (envelope glycoprotein (E), membrane (M), and capsid (C)) and seven nonstructural proteins (NS1, NS2a, NS2b, NS3, NS4a, NS4b, and NS5). Among them, E protein is the main structural protein with 55 kDa, which is a glycoprotein embedded in the viral membrane. It is known that E protein is not only a functional protein molecule that binds to receptors on the host cell membrane but also a major antigen, which can induce neutralizing antibody and host specific protective immunity [1–3]. As enveloped viruses, the DENVs enter the cells through receptor mediated endocytosis [4–7] and rearrange cell internal membranes to establish specific sites of replication [8–10]. As DENVs circulate between two hosts, humans and insects, they have to be adapted to replicate and infect both species. Recently there have been significant advances in understanding interactions of DENV with target cells such as dendritic cells (DCs), macrophages, vascular endothelial cells (VEC), and hepatocytes, and we would summarize receptors for DENVs on different cells identified in last several years in this review (Table 1).

## 2. DENV Receptors in DCs

After being bitten by an infected mosquito, immature DCs in the skin are believed to be the first target cells during DENV infection [11]. A C-type lectin mainly expressed by monocyte-derived DC [12, 13], named DC-specific ICAM 3-grabbing nonintegrin (DC-SIGN or CD209), mediates DENV infection. DC-SIGN is considered to be one of the most important receptors for DENVs [12–15]. Tassaneetrithep and his colleagues discovered that anti-DC-SIGN monoclonal antibodies could block DENV infection in DCs [13]. It was demonstrated biochemically that the interaction between DC-SIGN and DENV occurred through high-mannose N-linked glycans present in the viral envelope glycoproteins [16, 17]. Alen and his colleagues demonstrated that various carbohydrate-binding agents (CBAs) could block the replication of DENV1–4 in Raji/DC-SIGN+ cells as well as monocyte-derived DC (MDDC) [18]. MDDC, isolated from human donor blood, may not represent all DC subsets *in vivo*, but they express DC-SIGN, which made MDDC susceptible for DENV [12]. However, anti-DC-SIGN-specific antibodies could profoundly, but not completely, inhibit DENV infecting MDDC and other DCs. Till now complete inhibition of DENV infection is not achieved, indicating that other entry pathways are potentially involved in DCs.

## 3. DENV Receptors in Monocytes/Macrophages 

As had been observed previously in the MDDC, the infection of macrophages such as mature MDMØ was also blocked by anti-DC-SIGN antibodies [13]. Tassaneetrithep and his colleagues found that THP-1 cells (human acute monocytic leukemia cell line) become susceptible to dengue infection after the transfection of DC-SIGN [13]. Therefore, DC-SIGN may be considered as a new target for dengue infection in macrophages. However, only anti-DC-SIGN antibodies could not completely inhibit DENV infection in macrophages, indicating that there are other receptors mediating DENV entry into macrophages. Recently, it was shown that the mannose receptor (MR, CD206) was associated with DENV infection in macrophages [19]. In 2008, using enzyme linked immunosorbent assay (ELISA) and blot overlay assays, Miller et al. further demonstrated that MR could bind to all four serotypes of DENV and specifically to the E glycoprotein via its carbohydrate recognition domains. This binding was abrogated by deglycosylation of E protein [19]. A recombinant MR fusion protein (CRD4–7-Fc) was also shown to recognize E protein of DENV in ELISA and blot overlays, and the binding was inhibited by mannose, fucose, and EDTA [19]. Expression of recombinant MR on the surface of NIH3T3 cells conferred DENV increased binding and human MR antibodies could block this process in macrophages [19]. Pretreatment of primary human monocytes with Th2 cytokines such as interleukin IL-4/IL-13, which upregulated MR expression, could cause increase in their susceptibility to DENV infection *in vitro* [19]. All the above strongly suggest that MR is a novel functional receptor contributing to DENV infection in macrophages. However, it was shown that single antibody to either MR or DC-SIGN could not completely inhibit DENV infection while the combination of anti-DC-SIGN and anti-MR antibodies (CD206) was even more effective in inhibiting DENV infection in this kind of cells [19], indicating that several molecules may be involved in the process of DENVs entry into macrophages.

More recently, it was reported that C-type lectin domain family 5 member A (CLEC5A) contributed substantially to the mortality associated with DENV infection by triggering excessive macrophage activation and blockade of CLEC5A improved survival in mice [20]. Both human and mouse CLEC5A have been reported to bind to DENV, and the interaction was inhibited by fucose and mannan in vitro. Further studies showed that the CLEC5A-virus interaction triggered macrophage activation with a marked proinflammatory cytokine release through the associated adapter molecule DNAX-activating protein (DAP12) [20]. In addition, heat shock protein 90 (HSP90) and HSP70 have been identified as part of a receptor complex required for DENV entry and as CD14-independent cell surface functional receptors for lipopolysaccharide (LPS) in human monocytes/macrophages [21]. Interestingly, it has been reported that DENV infection was inhibited by bacterial LPS in human monocytes [22]. And also, Chen et al. found that the “binding” of LPS to CD14 was critical for DENV attachment and/or entry in macrophages [23]. About the phenomenon, Jorge Reyes-Del Valle and his colleagues offered an explanation: when monocytes were incubated with LPS prior to DENV infection, HSP90 and HSP70 were clustered around CD14, which prevented them from interacting with DENV [24], further implying an importance of HSP90 and HSP70 in the entry of DENV into monocytes/macrophages. 

## 4. DENV Receptors in Human VECs 

The endothelium is the primary fluid barrier of the vasculature, and the edema or hemorrhage seen in DHF/DSS is mainly due to changes in permeability of VEC induced by DENV infection. But the involvement of DENV receptors on VEC have not been revealed completely. One report, using a continuous ECV304 cell line, suggested that DENV interacted with three undefined cellular proteins [25]. However, these interactions have not been confirmed further in primary human VECs [26–28]. Lately, Dalrymple and Mackow found that DENV efficiently and productively infected human VECs via the interaction with heparan sulfate on glycosaminoglycan, heparan sulfate, as a nonspecific receptor molecule responsible for DENV attachment in several cell lines [22, 29]. Heparan sulfate is expressed in almost all cell types and is composed of alternating hexuronic acid/D-glucosamine disaccharides, which contains different degrees and patterns of sulfation, forming a linear chain with a remarkable diversity in length and structural complexity. The contribution of heparan sulfate to DENV entry has been shown by (i) a significant decrease in the binding capacity of DENV after enzymatic removal of heparan sulfate [30–34], (ii) a dose-dependent binding inhibition, which was only observed in heparin-pretreated mammalian cells, but not insect cell lines [31, 32, 35–37] suggesting that heparan sulfate as receptor for DENV was limited to mammalian cells, and the initial interaction (binding) between heparan sulfate and DENVs was likely influenced by the target cell types and viral serotypes [34], and (iii) an obvious decrease in virus binding to a mutant target cell lacking heparan sulfate expression [33, 37]. Interestingly, it was also demonstrated that DENV could bind specifically to immobilized heparin and both heparin and heparan sulfate ligands blocked DENV infection [33]. These findings were consistent with previous reports in which heparan sulfate proteoglycans (HSPGs) had been shown to mediate DENV attachment to Vero E6 cells and hepatocyte cell lines [22, 30, 33, 36]. Additionally, it was reported that purified E protein domains of DENV could interact with heparan sulfate [22, 38, 39], and VEC could not be infected by DENV after treatment with heparinase III, which cleaves both heparin and heparan sulfate side chains from cell surface HSPGs [29]. Together, all above results suggest that HSPGs were important receptors of DENV on VEC. However, there are some discrepancies. For example, Mertens et al. found that syndecans and glypicans were the most abundant HSPGs on cell surfaces, with syndecan-3 and glypican-1 being highly expressed on VEC, but syndecan antibodies failed to block DENV infection of endothelial cells [40, 41], indicating, other moleculars may act as receptor or coreceptor for mediating DENV entry into endothelial cells. In addition, Zhang and his colleagues found that high expression of integrin *β*3, which colocalized with dengue antigen, was observed in human microvascular endothelial cells 1 (HMEC-1) after dengue infection [42]. And about 90% of virus entry was inhibited when the expression level of integrin *β*3 was downregulated by RNA interference, indicating that DENV infection could induce upregulating expression of integrin *β*3, and integrin *β*3 was required for DENV entry into HMEC-1 [42]. Therefore, integrin *β*3 may be considered as a new target for dengue infection.

## 5. DENV Receptors in Hepatocytes

In severe cases of dengue, the impact of the DENV on liver function is prominent as shown by hepatomegaly and elevated serum levels of liver enzymes. Although the nature of the target cells for DENV in the liver is somewhat unclear, several studies based upon autopsy specimens have suggested the involvement of both hepatocytes and Kupffer cells [43–45]. Thepparit and Smith [46] identified the 37/67 kDa high-affinity laminin receptor as a DENV1 receptor expressed by HepG2 cells, a human hepatoma cell line, using a combination of virus overlay protein binding assay (VOPBA) and mass spectroscopy. The study also indicated that there was an association between the 37/67 kDa high-affinity laminin receptor protein and other glycoproteins at the cell surface, including the DENV low-affinity binding molecule heparan sulfate and the prion protein, suggesting that DENV receptor might be a complex consisting of those three proteins: heparan sulfate, the 37/67 kDa high-affinity laminin receptor, and prion protein [47]. Additionally in 2004, Jindadamrongwech and Smith identified the 78 kDa band for DENV2 as the glucose-related protein, GRP78 (BiP) on membrane extracts of HepG2 [48]. Pretreatment with anti-GRP78 antibodies resulted in a partial inhibition of DENV2 infection suggesting that additional receptor elements were involved in the entry process of DENV. In 2007, Cabrera-Hernandez and coworkers again noted a modest but definite inhibition of DENV2 entry into HepG2 cells in the presence of specific antibody directed against GRP78 [49]. The reproducible inhibition about 40% of the viral wild-type entry clearly demonstrated that GRP78 acted as at least a minor receptor in DENV internalization [49]. Moreover, it was reported that liver/lymph node-specific ICAM-3-grabbing integrin (L-SIGN) [50], homolog of DC-SIGN, expressed on liver sinusoidal endothelial cells as well as a subset of endothelial cells in the paracortex zone of lymph nodes, had the ability to bind to DENVs [51, 52]. And its expression in THP-1 cells induced susceptibility to DENV infection [53]. Specific antibodies against L-SIGN could subsequently block the acquired susceptibility. The L-SIGN-dependent DENV infection of THP-1 cells offered an intriguing possibility for the participation of L-SIGN in DENV infection [49].

## 6. Fc Receptors

Generally, DENV infection can induce subtype-specific humoral and cellular immune responses. If a secondary infection is caused by another serotype of DENV in the same individual, the preexisting antibodies will mediate virus infecting monocytes more efficiently. The outcome may be an increase in the viral replication and a high risk of severe dengue. This situation is referred to as antibody-dependent enhancement (ADE) of DENV infection. One possibility explaining this phenomenon is that in secondary infections, the virus may enter cells through the primary receptor(s) or it may also form immune complexes with preexisting nonneutralizing antibodies and interact with an alternative receptor, such as the immunoglobulin G (IgG) receptor (Fc gamma receptor, Fc*γ*R), which exists in Fc*γ*R-bearing cells including monocytes/ macrophages [54, 55]. By this process, the antibody-virus complexes may increase the ability of the virus to bind to and internalize into host cells, leading to maximum productive infection, that is, ADE of infection.

## 7. DENV Receptors on Mosquito Cells 

Generally more is known about the detail of DENV replication cycle in mammalian cells as compared with that in mosquito cells. An *Aedes albopictus* mosquito cell line (C6/36) was frequently used for almost all studies associated with DENV receptors in host of mosquito during recent years. In the earlier study, Salas-Benito and Del Angel [56] identified two membrane proteins about 40 and 45 kDa as DENV4 binding molecules expressed on the surface of C6/36 cells. Further study certified that the 45 kDa protein definitely was a DENV receptor protein and may be immunologically related to Hsp 90 [57]. Using the same method, Munoz and his group [58] identified two proteins of 67 and 80 kDa on C6/36 cells as putative DENV 2 receptor proteins. Following work found that these two proteins (67 and 80 kDa) acted as receptors for all four serotypes of DENVs [59]. In 2006, Sakoonwatanyoo and his colleagues identified two common bands of approximately 50 and 100 kDa. The protein of 50kDa could bind with DENV2, 3, and 4 and was supposed as laminin binding homologue that might play important roles in the internalization of DENV3 and DENV4 to C6/36 cells [60]. The band of 100 kDa could bind with DENV4 [61]. In 2010, Kuadkitkan indicated that prohibitin was specific for DENV2 in C6/36 cells, additionally shown to be significantly colocalized with E protein of DENV2, suggesting that the association of prohibitin-DENV2 interaction might be a multifunctional interaction occurring at several stages during the virus replication cycle [62]. In the same year, Paingankaret and his colleagues proposed a model for DENV2 entry and transport in mosquito cells: prohibitin, possibly in complex with an ATP synthase, Hsp70, actin, ava-1, and tubulin *β* chain, might serve to concentrate the virus particle at the cell membrane and activate a signal transduction pathway during infection, indicating that DENV2 may exploit an array of housekeeping molecules for its entry in C6/36 cells [63]. 

## 8. Others

The receptors used by flaviviruses are very complicated molecules. In addition to that mentioned above, recent studies have shown that the plasma membrane contains numerous microdomains, which are essential for cellular functions and are involved in viral infection. These lipid microdomains, also known as lipid rafts, were characterized by detergent insolubility, light density, and enrichment for cholesterol, glycosphingolipids, and GPI-linked proteins [24]. Cholesterol had a strong promoting effect on membrane binding and trimerization of DENV E protein [64]. To investigate the significance of lipid raft integrity for DENV entry, Jorge Reyes-Del Valle et al. [24] tested the infectious ability of DENV to human peripheral monocytes/macrophages pretreated with a lipid raft disrupter, such as methyl-cyclodextrin (MCD), an agent that depleted the cholesterol from the cells. They found that MCD treatment could inhibit DENV infection in a dose-dependent manner, suggesting that raft integrity was involved in DENV infection by clustering its receptor complex, which associated with membrane microdomains. Additionally, treatment with raft-disrupting drug could cause a significant inhibition in DENV infection, indicating that rafts may be a site for virus entry and thus had a profound impact on pathogenicity [24]. 

In summary, the receptors used by flaviviruses may defer very much, depending on cell types and viral serotypes [61]. Many findings strongly suggested that DENV probably bound to multiple molecules that might form complexes on host cells and that DENV used specific combinations of receptor candidates to enter different types of cells. Elucidation of the molecular mechanisms underlying the interaction of DENV with receptor(s) in humans and mosquitoes is not only essential for the understanding of dengue pathology but also crucial for the development of effective new therapies for treatment of dengue disease. Further investigations for understanding the nature of DENV receptor complex are required.

## Figures and Tables

**Table 1:** Dengue virus receptors found in different types of cells.

Cell types	Receptors
DC	DC-SIGN/L-SIGN
Monocyte/macrophage	DC-SIGN, MR, CRD4–7-Fc, CLEC5A, HSP90/HSP70, CD14-associated protein, and Fc*γ*R
VEC	Heparan sulfate, HSPGs, and integrin *β*3
Hepatocyte	Heparan sulfate, 37/67-kDa high-affinity laminin, prion protein, GRP78, and L-SIGN
C6/36 cell	HSP90/HSP70, 40/45 kDa membrane proteins, 50, 67, 80, and 100 kDa proteins, and tubulin-like protein
